This article has been retracted.

# Three-Dimensional Optimization Development and Regulation of Land Space Based on Spatial Equilibrium Model

**DOI:** 10.1155/2022/2933686

**Published:** 2022-03-27

**Authors:** Guoliang Zhai, Haibo Wang, Yulu Zhai

**Affiliations:** ^1^School of Architectural Engineering, Zhengzhou University of Industrial Technology, Zhengzhou 451150, Henan, China; ^2^School of Civil and Architectural Engineering, Anhui University of Science & Technology, Huainan 232001, Anhui, China; ^3^School of Landscape Architecture, Shangqiu University, Shangqiu 476000, Henan, China

## Abstract

The territorial space development pattern of the target construction should be able to help the full circulation and optimal allocation of social elements and resources, the society in the region is relatively fair, the development opportunities and welfare of people are equal, and the development of people, society, economy, and environment is coordinated and sustainable. This article aims to develop and control the three-dimensional optimization of the land space based on the spatial equilibrium model. This article first analyzes and introduces the spatial equilibrium model, then constructs an evaluation index model for the suitability of territorial spatial three-dimensional optimization development, and determines the index weights for the suitability of territorial spatial three-dimensional optimization development. Then, it analyzes the supply-demand relationship of the three-dimensional optimization development of the territorial space, discusses the imbalance of the supply and demand of the territorial service space, and finally summarizes the overall characteristics of the supply and demand of the three-dimensional optimization development of the territorial space based on the spatial equilibrium model. The research results show that under the conditions of rapid development, some development zones represented by the High-tech Zone in City B are seriously inadequate for industrial land use. In 2020, the proportion of industrial land in the high-tech zone of City B will exceed 17.69% of the 2015 plan. The demand for production space in the development zone is greater than the supply, which will inevitably bring certain pressure to industrial transformation.

## 1. Introduction

Territorial space is an ideal home for people to survive and thrive. However, due to the acceleration of the construction of modern urban projects, the total population of the city is expanding day by day, and the scale of urban construction and development is also expanding. In the past few decades, the area of built-up areas in small cities and towns has expanded by an average of about 113%, while the scale of urban population construction has increased by about 59%. The status quo of an extensive expansion of urbanization projects and the occupation of high-quality arable land has become more and more prominent, and the contradiction between the expansion of urban production space and living space and the natural ecological environment has become more and more prominent. The history of modern urbanization projects in Western countries has proven that when the urbanization rate reaches 30%, there will be some urban project construction problems, so the city plan will be implemented. However, when the urbanization rate reaches 50%, social problems such as uncoordinated urban and rural development, unbalanced regional development, conflicts with economic and social development concepts, and environmental and social issues will arise. At this time, urban space planning has emerged as a key tool to promote sustainable development.

The land space development layout refers to the distribution of people's entire social business activities in the geographical space. A scientific and reasonable land space development layout can promote the rational circulation and optimal distribution of the entire social business elements. The development opportunities of each person in the space and the community's interest levels are fair, and the coordination of the national economy, interests, overall population resources, and environmental protection has been achieved. The rapid economic and social development and the continuous inflow of a large number of people have caused various problems such as congestion of living space, pollution of natural resources, continuous shortage of high-quality land around cities, and uneven environmental conditions for regional development. This paper aims to develop and control the three-dimensional optimization of land space based on the spatial equilibrium model, so as to provide an important theoretical basis for the development of the whole society and natural ecology.

According to the research progress at home and abroad, different scholars also have a certain degree of cooperative research on spatial equilibrium models and three-dimensional optimization of territorial space: Wan and Jin proposed a new model calibration verification strategy based on a spatial equilibrium model, which combines multiple time ranges, so that the predictive ability of the model can be empirically tested. Model verification through forward and backward prediction is helpful to verify the stability of model parameters and predict the recursive equilibrium framework. The proposed modeling strategy sets a new standard for verifying the recursive equilibrium model [1]. Kurichev has developed a new model of spatial balance in MA, which includes three modules: (1) the spatial equilibrium model of MA labor and housing market, (2) the dynamic equilibrium model of Malian immigration and housing construction, and (3) the distribution model of housing construction in various regions [2]. Takayama et al. researched and developed a spatially computable equilibrium model that takes into account the agglomeration economy and the mobility of production factors. It also introduces parameter estimation and calibration procedures and a method to obtain stable equilibrium with changes in structural parameters. Using these methods, the study quantified the impact of reduced trade costs in Japan and clearly described the characteristics of the developed model [3]. Ishikura and Kimura constructed a spatially computable general equilibrium model characterized by international transportation corridor regions. The model clearly regards export industries and import industries as the transportation service industries required for international trade. By introducing the concept of iceberg transportation cost, the domestic interregional transportation system is clearly modeled [4]. Taking the Yunnan-Guizhou Plateau as an example, Xu et al. proposed a comprehensive ecological risk assessment method to provide technical reference for land-use optimization. In order to ensure the sustainable use of regional land resources, the following suggestions are made: (1) change the extensive and inefficient use of land and promote the economic and intensive use of flat land; (2) promote industrial projects and the construction of hillside cities according to local conditions; (3) strengthen ecological environment protection, promote the development and utilization of gentle slope wasteland, prevent erosion, and avoid geological disasters [5]. Sahebgharani developed a new metaheuristic algorithm called Parallel Particle Swarm and then compared the output of the newly developed algorithm with the output of the genetic algorithm. The results show that the output achieved by the two algorithms is better than the current land use distribution status. Therefore, this method can be used as a tool in the hands of urban planners and decision-makers to support the planning of land use processes [6]. Dan et al. carried out an evaluation of the suitability of urban and rural construction land development, calculated the critical threshold of urban and rural construction land, calculated the abundance of urban and rural construction land, and compared it with the current urban and rural construction land. The research results help to clarify the relationship between the current development status and the reasonable development status and provide a basis for the formulation of the fine management of urban and rural construction land and the optimization and control policy of the spatial pattern [7]. Rezk et al. compare PSOGWO with other state-of-the-art methods. The obtained results confirm that the smallest RMSE value is achieved with PSOGWO for all case studies compared to the PSO and GWO optimizers. PSOGWO achieves an almost perfect agreement between estimated and experimental datasets [8]. Hans and Kaur proposed a binary version of the MVO algorithm with two main purposes: first, to remove redundant and irrelevant features from the dataset, and second, to achieve better classification accuracy. The proposed binary version uses the concept of a transition function to map successive versions of the MVO algorithm to its binary version [9]. Borhani analyzes the flight network structure in air transportation by using the multiobjective genetic algorithm of geographic information system (GIS), which is used to optimize the topology structure of Iran Airlines to reduce the number of routes and the aggregation of passengers. The proposed multiobjective genetic algorithm (MOGA) was tested and evaluated on data from the Iranian aviation industry in 2018 as an example of practical application for designing the topology of the Iranian airline [10]. However, these scholars did not combine the spatial equilibrium model with the three-dimensional optimization of the territorial space to explain the problem but only unilaterally explored their significance.

The innovation of this article is reflected in the following. (1) It analyzes and introduces the spatial equilibrium model, constructs an evaluation index model for the suitability of three-dimensional optimization and development of land space, and determines the index weight of the suitability of three-dimensional optimization and development of land space. (2) Then, it analyzes the supply and demand relationship of three-dimensional optimal development of land space and discusses the imbalance between supply and demand of land service space. (3) Finally, the general characteristics of supply and demand for three-dimensional optimal development of land space based on the spatial equilibrium model are summarized.

## 2. Three-Dimensional Optimization Development and Control Method of Land Space Based on Spatial Equilibrium Model

### 2.1. Spatial Equilibrium Model

The idea of spatial balance is the application of general equilibrium theory to the regional economy. In fact, it is not equivalent to “equality” in economics. The concept of “space” in Earth science refers to an abstract organism that contains certain social, economic, ecological, and other resources. It is also an activity carrier, including natural and social attributes [11, 12]. We should correctly understand the unity of the natural and social attributes of space in order to better understand the nature of space. “Balance” originates from the concept of Western economics, which means equality, including quantity and state. When the quantity supplied is equal to the quantity demanded, the price should reach equilibrium. In short, territorial balance can also be understood as the coordination between the development of space economic activities and the ability to provide territorial locations in a given region [13].

The supply capacity of different regions depends on the social, economic, ecological, and other resources of the region, and the development capacity depends on the supply capacity of the region [14]. In the context of economic globalization, trade and division of labor between regions cannot meet the space needs in a given region but can only be provided by other regions [15]. In this regard, the regional balance is based on the overall balance of supply and demand and the orderly division of production and ecological models into different regions [16].  Figure 1 shows the operating network structure of the big data platform for land and space planning. With the rapid development of related information technology in recent years and the introduction of related big data technology, new changes have gradually appeared in related land and space planning. As one of the important databases affecting national development and related policy planning, the planning of land space has an important impact on the relevant macrocontrol and sustainable development of the country. At the same time, it is also an important basis for affecting the correctness, accuracy, and scientificity of relevant decisions, an important factor to change the country's current state of land and space resource utilization, and an important measure to improve the efficiency of related land and resource utilization. On the basis of the above, territorial development and its supply capacity should be coordinated with each other [17]. If the development demand intensity of territorial development is not coordinated with its supply capacity, it will lead to incoordination of the region's society, economy, resources, and environment, leading to territorial imbalance [18].

In short, the concept of territorial balance in land use can be understood as that in a specific area, human beings are pursuing economic development [19]. The coordinated behavior between the economic activities of land use and the natural distribution of land resources enables the spatial development mode of land use to achieve territorial balance, maximizes the overall benefits of all aspects of society, and ensures that land use reaches the goal of sustainable development [20]. In short, when the territorial supply capacity is equivalent to the intensity of territorial development and utilization, regional territorial development reaches a territorial balance. The degree of coordination between the territorial supply capacity and the intensity of territorial use and development is the degree of balance of territorial use in the region [21]. If the regional supply capacity of soil exceeds the development intensity of land use, it means that the regional development of land use is insufficient (spatial imbalance). If the regional supply capacity of soil is equivalent to the intensity of land use and development, the regional use and development model should achieve a geographical balance. When the regional land supply capacity is lower than the development intensity of land use, the land-use area will be overexploited (spatial imbalance) [22].  Figure 2 shows the network design of the land and resources system based on the Internet terminal.

### 2.2. Constructing an Evaluation Index Model for the Suitability of Territorial Spatial Three-Dimensional Optimization Development

The suitability of theoretical research on territorial spatial structure refers to the natural carrying capacity of territorial spatial structure (including soil, geological environment, and natural resources), the development attributes of the community's economic environment, and its future development capabilities, to study in depth and determine the suitability of the territorial spatial structure to the established function, and whether it is suitable for development constraints [23].

#### 2.2.1. First-Level Evaluation Model

The first-level evaluation model *A*_*mn*_(*m*=1,2,3; *n*=1,2 …, *l*) is built on the second-level index system *A*_*m*_, that is, the evaluation model of *A*_*mn*_⟶*A*_*m*_. The construction of the first-level evaluation model is based on the specific evaluation index *A*_*mn*_.  Figure 3 shows the general equilibrium theoretical model.

  Hypothesis: the area to be evaluated includes Q area units, and the measured value of the n-th index *A*_*mn*_ in the second-level evaluation index set *A*_*m*_ on the k-th area unit is *A*_*mn*_^*k*^(*k*=1,2,…, *q*) [24].

Note

(1) $$\begin{array}{c} A_{mn}^{\max}=\max\;A_{mn}^{k},\\ A_{mn}^{\min}=\min\;A_{mn}^{k}. \end{array}$$

If *A*_*mn*_ is the bigger the better, that is, the positive index, let

(2) $$\begin{array}{c} u_{mn}^{k}=\frac{\left[A_{mn}^{k}-A_{mn}^{\min}\right]}{\left[A_{mn}^{\max}-A_{mn}^{\min}\right]}. \end{array}$$

If *A*_*mn*_ is the smaller the better, that is, the negative index, let

(3) $$\begin{array}{c} u_{mn}^{k}=\frac{\left[A_{mn}^{\max}-A_{mn}^{k}\right]}{\left[A_{mn}^{\max}-A_{mn}^{\min}\right]}. \end{array}$$

Obviously, for the evaluation index *A*_*mn*_, *u*_*mn*_^*k*^ is the degree of subordination of the k-th regional unit in the “suitability of land and space development” [25]. In this way, the following membership matrix can be obtained:

(4) $$\begin{array}{c} U_{m}=\left|\begin{array}{ccccc} u_{m1}^{1} & u_{m1}^{2} & u_{m1}^{3} & \ldots & u_{m1}^{q}\\ u_{m2}^{1} & u_{m2}^{2} & u_{m2}^{3} & \ldots & u_{m2}^{q}\\ u_{m3}^{1} & u_{m3}^{2} & \begin{array}{c} u_{m3}^{3}\\ \ldots \end{array} & \ldots & u_{m3}^{q}\\ u_{ml}^{1} & u_{ml}^{2} & u_{ml}^{3} & \ldots & u_{ml}^{q} \end{array}\right|. \end{array}$$

In the second-level evaluation index combination *A*_*m*_, if the weight of each rating index is allocated as *H*_*m*_=(*h*_*m*1_, *h*_*m*2_,…, *h*_*ml*_), the first-level evaluation index result can be obtained by the following transformation formula:

(5) $$\begin{array}{c} R_{m}=\left(r_{m}^{1},r_{m}^{2},\ldots ,r_{m}^{q}\right)=H_{m}*U_{m}. \end{array}$$

In the formula, *r*_*m*_^*k*^ (*k*=1,2,…, *q*), for the second-level evaluation, is the degree of subordination of the k-th regional unit to the “suitability of land and space development.”

#### 2.2.2. Secondary Evaluation Model

In the first-level evaluation index set A, if the weight distribution of the evaluation index sets at all levels is *R*=(*r*_1_, *r*_2_,…, *r*_*l*_), then based on the calculation of the first-level evaluation model, the second-level evaluation conclusion, that is, the comprehensive evaluation conclusion is

(6) $$\begin{array}{c} R=\left(r^{1},r^{2},\ldots ,r^{q}\right)=R*U. \end{array}$$

In the formula, *U*=(*R*^1^, *R*^2^,…,*R*^*q*^)^*U*^ and *r*^*k*^(*k*=1,2,…, *q*) are relative to the evaluation index system A, which is the degree of subordination of the k-th regional unit to the “suitability of land and space development” [26].

After arranging *r*^*k*^(*k*=1,2,…, *q*) from the largest to the smallest, we can get the ranking of the advantages and disadvantages of the comprehensive evaluation of the suitability of each area or unit land space development to be evaluated [27].

### 2.3. Determining the Weights of the Suitability Index for the Three-Dimensional Optimization and Development of Territorial Space

The coefficient of variation method can be used to determine the weight of indicators for the suitability of territorial development. The coefficient of variation is a more objective weighting method. It directly uses the information involved in each index and then obtains the weight of each index through statistics.

The first step is data standardization. The standard deviation standardization method is used to standardize the research data, and according to the indicator trend, it is divided into positive indicators and negative indicators for standardized management.

(1) Positive index, that is, the larger the index value, the better. Its standardized model is
  (7) $$\begin{array}{c} j_{mn}=\frac{A_{mn}-A_{\min}}{A_{\max}-A_{\min}},\\ S_{mn}=\frac{s_{mn}-\min\left(s_{n}\right)}{\max\left(s_{n}\right)-\min\left(s_{n}\right)}. \end{array}$$
(2) Negative index, that is, the smaller the index value, the better. Its standardized model is
  (8) $$\begin{array}{c} j_{mn}=\frac{A_{\max}-A_{mn}}{A_{\max}-A_{\min}},\\ S_{mn}=\frac{\max\left(s_{n}\right)-s_{mn}}{\max\left(s_{n}\right)-\min\left(s_{n}\right)}. \end{array}$$

The second step is to calculate the average $\bar{s_{m}}$ and standard deviation *φ*_*m*_ of each index data after the standardization process. The calculation formula is as follows:

(9) $$\begin{array}{c} \bar{s_{m}}=\frac{1}{l}\sum_{n=1}^{l}s_{mn}n=1,2,3\ldots l,\\ \varphi_{m}=\frac{1}{l-1}n=1\sum_{n=1}^{l}{\left(s_{mn}-\bar{s_{m}}\right)}^{2}n=1,2,3\ldots l,\\ T_{mn}=\frac{S_{mn}}{\sum_{m=1}^{l}S_{mn}}. \end{array}$$

The third step is to calculate the coefficient of variation *d*_*m*_ of each index. The calculation formula is as follows:

(10) $$\begin{array}{c} d_{m}=\frac{\bar{s_{m}}}{\varphi_{m}}\;m=1,2,3\ldots l,\\ R_{n}=-j\sum_{m=1}^{l}T_{mn}\ln\;T_{mn}, \end{array}$$

among

(11) $$\begin{array}{c} j=\frac{1}{\ln\;l}. \end{array}$$

The fourth step is to calculate the weight *H*_*m*_ of each indicator:

(12) $$\begin{array}{c} H_{m}=\frac{d_{m}}{\sum_{m=1}^{l}d_{m}m=1,2,3\ldots l},\\ H_{n}=\frac{1-R_{n}}{\sum_{m=1}^{l}\left(1-R_{n}\right)}. \end{array}$$

The weighted sum method is used to calculate the suitability of land and space development. The calculation formula is

(13) $$\begin{array}{c} R=\sum_{m=1}^{l}H_{m}A_{m}. \end{array}$$

In the formula, R is the suitability of land space development, *H*_*m*_ is the weight of the m-th index, and *A*_*m*_ is the standardized value of the m-th index.  Figure 4 shows the research technology roadmap for the balanced development of land space.

## 3. Experimental Results of Three-Dimensional Optimization Development and Regulation of Territorial Space Based on the Spatial Equilibrium Model

This paper aims to develop and control the three-dimensional optimization of land space based on the spatial equilibrium model, so as to provide an important theoretical basis for the development of the whole society and natural ecology. The supply and demand relationship of three-dimensional optimal development of land space is analyzed and researched. At the same time, the significant reasons for the imbalance between supply and demand of land service space are explored, and the overall characteristics of supply and demand for three-dimensional optimal development of land space based on the spatial equilibrium model are analyzed.

### 3.1. Supply and Demand for Three-Dimensional Optimized Development of Territorial Space

The strong demand for total production space in the early development zone has led to an excessively large proportion of industrial land, and the problem of spatial homogeneity has slowly emerged. After entering the transition period, its total demand began to gradually decline, resulting in a decline in the proportion of industrial land, and space transformation is imminent.

#### 3.1.1. Reduction in Total Demand

With the gradual unfolding of the “two retreats and three advances” process of some industrial land in the development zone, the demand for production space in the development zone has turned from strong to weak, the growth rate of total demand has slowed, and the transformation of production space is quietly unfolding. Statistics show that before the transition period, the average proportion of industrial land in the four development zones in the Yangtze River Delta reached 42%, which was nearly 17% higher than the national standard. After the transition period, the average annual growth rate of industrial land was only −1.02%. In particular, the proportion of high-tech zones in City B has dropped from 59.78% in the previous period to 49.21%, an average annual decrease of about 3.43%, as shown in Figure 5.

#### 3.1.2. Supply is Still Scarce

Compared with the expansion of demand for production space, the total space supply of the development zone is relatively insufficient. According to statistics in the past five years, under conditions of rapid development, some development zones represented by the High-tech Zone in City B are seriously in short supply of industrial land. In 2020, the proportion of industrial land in the high-tech zone of City B will exceed 17.69% of the 2015 plan, as shown in Figure 6. It can be seen that the demand for production space in the development zone is greater than the supply, which will inevitably bring certain pressure to industrial transformation.

The initial goals of the development zone are different: the economic and technological development zone mainly uses foreign capital to develop an export-oriented economy; the high-tech industrial development zone is mainly engaged in scientific and technological research and industrial development. In order to pursue economic benefits, development zones often take the initiative to attract foreign investment, carry out foreign industrial transfers, and pay more attention to “OEM production” rather than “high-tech industrialization of research and development.” This distorted the initial development goals of the two types of development zones, made the direction of industrial development apparently converged, and led to the homogenization of the structure of production space demand. With the increase in the number of overseas financing companies, its impact on the development zone has further deteriorated. The survey shows that from 2006 to 2018, the impact of foreign-funded enterprises on the high-tech sector has shown a clear upward trend year by year, with the overall contribution rate rising from 3.01% to 60.2%.

### 3.2. Significant Imbalance between Supply and Demand of Territorial Service Space

Since the establishment of the development zone, the supply and demand of the service space in the development zone has been cleared out of balance. In particular, the following problems have arisen in terms of total space and layout. The increase in the residential population, the improvement of the industrial structure, and the gradual development of the service industry in the development zone have promoted the total demand for service space from low to high, but the space supply is obviously lagging behind the demand. At the same time, the demand structure of a single service area also affects the further development of the development zone.

#### 3.2.1. Demand from Low to High

The demand for service space in the development zone is gradually increasing, but the growth rate is slow and the total amount is not large. According to statistics, after years of development in the four development zones in the Yangtze River Delta, the proportion of land used for public service facilities has continued to rise, with an average annual growth rate of 0.41%. Due to advanced planning, the average annual growth rate of land use in City A's industrial parks is even as high as 1.35%, as shown in Figure 7.

#### 3.2.2. Long-Term Supply Lag

In the short term, the supply of service space in the development zone has been unable to meet the growing demand, and it appears to be a long-term lag. Statistics found that the public service land in the seven major development zones in the Yangtze River Delta was overbuilt by an average of nearly 2.35% compared with the earlier planned. Among them, from 2004 to 2008, the construction of public service land in the economic and technological development zone of city F exceeded 4% in four years. As shown in Figure 8, it can be seen that the supply of service space has been stagnant.

#### 3.2.3. Imperfect Demand Structure

In terms of service space, the demand combination of residential service space and product service space is not yet perfect. On the one hand, due to the large number of industrial population, citizens, and primary and secondary school students in the economic development zone, the scale of residential land is rapidly expanding, and the demand for production and residential service space is increasing, but the function is still relatively single; on the other hand, industrial enterprises pay more attention to the processing and production of physical objects and have less demand for production service space. According to the survey, the land for public service facilities in the two development zones in the Yangtze River Delta is relatively single, mainly for commercial finance and education; residential service space is mainly commercial facilities such as commerce and retail, and production service space is mainly higher education facilities. Land for culture, entertainment, sports, and scientific research is relatively scarce, as shown in Table 1.

### 3.3. The Overall Characteristics of Supply and Demand for the Three-Dimensional Optimized Development of Territorial Space Based on the Spatial Equilibrium Model

Through the above analysis of land space supply and demand, it is not difficult to see that the contradiction between the scarcity of land space supply and the diversity of demand will lead to an imbalance in the spatial proportional structure and layout structure of the development zone. In general, the supply and demand of land space has the following two characteristics.

#### 3.3.1. Supply Lags Behind Demand in Stages

The total territorial supply of the development zone is gradually lagging behind the demand, and there is a gap in the territorial proportion structure.

With the development and evolution of development zones, even the dominant attributes of space requirements are also changing. In the initial stage, as the only industrial zone, the development zone's demand for production space is completely dominant; during the growth period, with the rapid expansion of the development zone, the demand for production and living space dominates; after the end of the industrial structure transformation period, the demand for service space will become dominant, and the development zone will gradually move toward a mature stage of innovation and integration, as shown in Figure 9.

Compared with the evolution of space demand, space supply is passive and lagging, resulting in insufficient space supply and lack of space structure, resulting in low space efficiency and insufficient innovation capabilities in development zones, as shown in Table 2. Absence refers to the structural lack of functional space, which is usually manifested as a delay in space supply and an imbalance in internal structure.

In recent years, the territorial proportion structure of the development zone has been seriously inadequate. It is worth noting that the proportion of existing industrial land in the Yangtze River Delta Development Zone is too high, 2.3 times that of the Adlershof High-tech Industrial Development Zone; the proportion of public service land is too low, even less than 1/3 of the Adlershof development zone, as shown in Table 3.

#### 3.3.2. Periodic Deviation of Supply and Demand

The supply and demand of the regional arrangement of the development zone has the characteristics of periodic deviation. Specifically, in order to meet the space needs of advanced development, the development zone continues to promote a new round of land supply planning and adjustments. However, the space supply in the development zone still lags behind the demand, and there is a large gap between supply and demand. From the perspective of the change curve of land supply and demand in the development zone, there is a clear deviation in the overall space supply and demand of the development zone from the initial stage to the growth period; after entering the transition period, the deviation between supply and demand gradually decreases, as shown in Figure 10.

The deviation of space supply and demand will lead to the dislocation of the spatial layout structure of the development zone; that is, the function is broken and the layout of spatial elements is chaotic. The specific manifestation is the imbalance of the spatial structure, and the formation of industrial clusters is difficult; the details are shown in Table 4.

## 4. Discussion

The population policy under the functional differentiation of territorial space can be analyzed from two aspects: narrow policy and broad policy. Among them, the narrow policy mainly includes the population birth and migration policy, the purpose of which is to form a population layout that conforms to the land and space function planning, and the broad policy refers to the related supporting measures adopted for the smooth implementation of the narrow population policy. In terms of narrow policy, the content of population planning in regional planning should be readjusted. Under the positioning of territorial space function, the population capacity of each region should be accurately calculated, so that the regional population and the regional territorial space function positioning should be coordinated. For each type of region, we formulate differentiated population migration policies. For example, for regions with better development status, we should promote the localization of the immigrant population with fixed occupations and residences as soon as possible. As for regions with development potential, more migrants should be absorbed to protect the basic rights and interests of floating populations. For the population that needs to be relocated due to the functional positioning of the land and space, overall planning and guidance should be carried out on the basis of various supporting infrastructures and stable employment opportunities to protect their normal living conditions and rights. In terms of broad policies, first, we strengthen the protection of farmland ownership of farmers, and on the basis of economical use of farmland, we allow farmers to realize the greatest benefit of farmland use rights in the differential income. Second, we strengthen the supporting reforms of the social security system and raise the level of overall planning to promote the cross-regional flow of labor and population, and to promote the realization of the functional positioning of the land and space, combining the actual development of various types of regions, we promote the equalization of public services between regions. Since the basic goal of building a socialist society is to achieve common prosperity, promoting equalization of basic public services between regions is the basic requirement for building a people-oriented harmonious society and regional coordinated development.

## 5. Conclusions

Through empirical research on the Yangtze River Development Zone, it is found that insufficient supply of production and service space is often unable to meet diversified needs, which is manifested as a problem of insufficient supply. In-depth analysis shows that the contradiction between supply and demand in territorial development has its own unique reasons. In the process of construction and development, the negative effects of land policies, the drawbacks of economic transformation, and the blindness of site selection for construction projects will all lead to conflicts between land supply and demand. First, in the context of the land policy of “supporting land areas,” deceptive land transfer policies and lack of regulatory policies have led to a strong demand for industrial land, resulting in inefficient space development, controlling the real estate market, and effectively providing insufficient residential space. Second, in the context of economic transformation, the industrial structure in the development areas is backward, the employment structure and work knowledge structure are not perfect, and the atmosphere of innovation has not yet formed so that the supply and demand relationship between production and service space has not decreased. Third, the timing of project investment and construction is not coordinated, and the site selection is blind, resulting in a dislocation of the overall layout structure and stagnant land space reconstruction. This paper studies the three-dimensional optimization and development regulation of land space based on the spatial equilibrium model, in order to provide a realistic theoretical basis for the development of the whole society, national economy, and ecology.

## Figures and Tables

**Figure 1:** The operational network structure diagram of the big data platform for land and space planning.

**Figure 2:** System network design.

**Figure 3:** General equilibrium theoretical model.

**Figure 4:** Research technology roadmap.

**Figure 5:** Comparison of the growth of the proportion of industrial land in the four major development zones in the Yangtze River Delta.

**Figure 6:** Comparison of industrial land planning and built-up proportion of the seven major development zones in the Yangtze River Delta.

**Figure 7:** Comparison of the growth in the proportion of public service land in the four major development zones in the Yangtze River Delta.

**Figure 8:** Comparison of public service land planning and construction proportion of the seven major development zones in the Yangtze River Delta.

**Figure 9:** Leading demand space in different development stages of the development zone. Note: PS: production space; RS: residential space; SS service space.

**Figure 10:** Development zone land layout supply and demand curve. *Note.* D land layout demand; S land layout supply; M land layout perfection; As ∼ Ad, Bs ∼ Bd: deviation of supply and demand at different stages.

**Table 1:** The current composition of land for public service facilities in the high-tech zone of City A and the economic and technological development zone of City B (%).

Name	Administration	Business finance	Culture and entertainment	Physical education	Health care	Education and research	Business office mix
High-tech zone, City A	12.1	34.9	0.9	1.1	5.5	42.9	0.6
F city economic development zone	19.1	41.4	6.2	1.8	2.9	3.2	10.2
Average proportion	15.6	38.2	3.5	1.5	4.2	23.1	5.4

**Table 2:** List of the total supply and demand of land space in the development zone and the corresponding spatial ratio structure problems.

Serial number	Space type	Time	Supply and demand	Spatial proportion structure problem
1	Production space	3 months	Need < supply	Lack of agglomeration and low capacity
		9 months later	Need > supply	Excessive weight, inefficient development
2	Living space	3 months later	Need > supply	Housing is scarce and still vacant
3	Service space	3 months later	Need > supply	Service is scarce, center is missing
		3 months later	Need > supply	Low structure, lack of innovation
4	Overall space	3 months later	Need > supply	Lack of space, inefficient development

**Table 3:** Comparison of the current average proportion of land used in the seven major development zones in the Yangtze River Delta with other standards.

Name	Industry	Live	Public facilities	Green field
The average proportion of land used in the seven major development zones of the Yangtze River (%)	43.1	17.1	8.6	8.1
National construction land standard (%)	13∼24	18∼29	—	6∼16
Proportion of land used in the Adlersh of the development zone in Berlin, Germany (%)	19.1	10.2	24.7	21.2

**Table 4:** List of supply-demand relations and corresponding spatial structure issues in the development zone's territorial spatial layout.

Serial number	Space type	Time	Supply and demand	Spatial layout structure problem
1	Production space	3 months	Need < supply	—
		9 months later	Need > supply	Disorderly spread, inefficient operation
2	Living space	3 months later	Need > supply	Residence differentiation, separation of job and residence
3	Service space	3 months later	Need > supply	The layout is chaotic and the neighborhood is missing
		3 months later	Need > supply	Discrete space, not clustered
4	Overall space	3 months later	Need > supply	Dislocation of space, unbalanced structure

## Data Availability

No data were used to support this study.
